The article "Accumulative Quantization for Approximate Nearest Neighbor Search" was published in 2022. Journal: Comput Intell Neurosci.

# Accumulative Quantization for Approximate Nearest Neighbor Search

**DOI:** 10.1155/2022/4364252

**Published:** 2022-02-15

**Authors:** Liefu Ai, Yong Tao, Hongjun Cheng, Yuanzhi Wang, Shaoguo Xie, Deyang Liu, Xin Zheng

**Affiliations:** ^1^School of Computer and Information, Anqing Normal University, Anqing 246133, China; ^2^University Key Laboratory of Intelligent Perception and Computing of Anhui Province, Anqing Normal University, Anqing 246133, China; ^3^School of Electronic Engineering and Intelligent Manufacturing, Anqing Normal University, Anqing 246133, China

## Abstract

To further improve the approximate nearest neighbor (ANN) search performance, an accumulative quantization (AQ) is proposed and applied to effective ANN search. It approximates a vector with the accumulation of several centroids, each of which is selected from a different codebook. To provide accurate approximation for an input vector, an iterative optimization is designed when training codebooks for improving their approximation power. Besides, another optimization is introduced into offline vector quantization procedure for the purpose of minimizing overall quantization errors. A hypersphere-based filtration mechanism is designed when performing AQ-based exhaustive ANN search to reduce the number of candidates put into sorting, thus yielding better search time efficiency. For a query vector, a self-centered hypersphere is constructed, so that those vectors not lying in the hypersphere are filtered out. Experimental results on public datasets demonstrate that hypersphere-based filtration can improve ANN search time efficiency with no weakening of search accuracy; besides, the proposed AQ is superior to the state of the art on ANN search accuracy.

## 1. Introduction

Nearest neighbor (NN) search is fundamental and important in many applications, such as machine learning, image classification, content-based image retrieval, deep learning, feature matching [1], and image interpolating [2]. The goal of NN search is to find the closest vector whose distance to the query vector is the smallest among a database according to a predefined distance metric.

The natural solution is to perform exact nearest neighbor search, which is inherently expensive for large-scale collects and high dimensional vectors due to the “curse of dimensionality” [3]. This difficulty has led to the development of the solutions to approximate nearest neighbor (ANN) search. The key idea shared by ANN methods is to find the NN with high probability “only,” instead of probability 1 [4] by exhaustive search or nonexhaustive search based on index [5–7].

Hash-based nearest neighbor search methods map vectors from Euclidean space into hamming space, using binary codes to represent the vectors [8]. The similarity between vectors is measured by the hamming distance between the codes. Such methods include small binary code [3], spectral hashing [9], spherical hashing [10], hamming embedding [11], mini-BOF [12], and K-means Hashing [13]. These methods make it possible to store large-scale vectors in computer memory and perform nearest neighbor search efficiently. While promising, when the number of bits used for encoding vectors is fixed, the possible number of hamming distances is consequently fixed. Therefore, the discrimination of hamming distance is restricted by the length of code.

There are ANN search methods trying to resolve the nearest neighbor search problem with efficient quantization technology [14] by adopting Euclidean distance which owns better discrimination than hamming distance. As a typical work, product quantization (PQ) is firstly introduced into ANN search [4], where the vector space is decomposed into a Cartesian product of low-dimensional subspaces. A vector is represented by a short code composed of its subspace quantization indices. An asymmetric Euclidean distance is designed to accelerate the approximate distance computation between two vectors. It is proved to be superior to hamming distance in terms of the trade-off between accuracy and search time efficiency. A lot of PQ variants [15–23] are studied to improve the performance in different ways, such as optimized product quantization (OPQ) [16], product quantization with dual codebooks [19], Cartesian k-means [20], and Quarter PQ [21].

PQ assumes that each dimension component in vectors is statistically independent of each other, while this is not applicable enough for all real data. Contrast to PQ-based methods which partition vector space into several subspaces, another representative quantization research community mainly focuses on approximating a vector *v* by using the addition of *L* centroids *c*_*v*,*l*_ with each selected from one codebook (equal (1)). Then, the vector is represented by a short code composed of the indices of *L* selected centroids.

(1) $$\begin{array}{c} v\approx \sum_{l=1}^{L}c_{v,l}. \end{array}$$

The typical works include addition quantization [24] and composite quantization (CQ) [25]. CQ trains codebooks by introducing near-orthogonal constraint while addition quantization minimizes the quantization errors over each dimension during training codebooks. In contrast, residual vector quantization (RVQ) [26, 27] is a sequential multistage quantization technique consisting of several stage-quantizers. Except the first stage, the vectors used to train the stage-codebook are the residual vectors generated from the preceding stage-quantizer. Enhanced RVQ [28] improves the accuracy of approximating a vector by designing a joint optimization to reduce overall quantization errors during training codebooks. Based on RVQ, project residual vector quantization [29] improves the training efficiency by projecting vectors into low-dimensional vector space, while projection-based enhanced residual quantization [30] is based on enhanced RVQ.

In this paper, we propose an accumulative quantization method for ANN search to further improve search accuracy. This paper offers the following contributions:

1. Accumulative quantization is proposed to represent a vector as a sum of *L* partial vectors which are quantized by *L* codebooks, respectively. For this, each vector is firstly decomposed into *L* components of the same dimension as that of original one. Then, initial *L* codebooks are trained on those *L* partial vector sets independently. To improve the approximation power of codebooks, an optimization is introduced through minimizing the overall error between original vector and the vector reconstructed by accumulative quantization.
2. In the ANN search procedure, to gain good search accuracy, *R* search results are usually returned. Normally, whether exhaustive search or nonexhaustive search, the candidate vectors are sorted to get the *R* search results of high probability with the distance between candidates and the query vector. Then, the number of candidate vectors restricts the time efficiency of ANN search. Actually, given a query vector, its nearest neighbors only locate near the query in the vector space, so we proposed a hypersphere filtration strategy, which has simple but positive effect on improving search time efficiency. By constructing a hypersphere with each query vector as the center, only the candidates located in the hypersphere are put into sorting.

This paper is organized as follows: Section 2 presents accumulative quantization (AQ). An asymmetric distance with uniform scale quantization is described in Section 3.  Section 4 introduces a hypersphere-based filtering strategy and the combination with AQ-based exhaustive ANN search. The performance of our approaches and the comparisons with the state of the art are reported in Section 5. Conclusions are discussed in Section 6.

## 2. Accumulative Quantization

Given a vector *v*, accumulative quantization approximates the vector as the sum of *L* partial vector, where each partial vector is quantized with a pretrained codebook, as follows:

(2) $$\begin{array}{c} v=\sum_{l=1}^{L}v_{l}\approx \sum_{l=1}^{L}{\hat{v}}_{v,l}=\hat{v}. \end{array}$$

where ${\hat{v}}_{v,l}$ is the quantization output centroid selected from the *l*th codebook. Then, vector *v* is represented by the *L*-tuple indices of centroids corresponding to ${\hat{v}}_{l,v}$.

The quantization accuracy can be measured by the difference between *v* and its reconstructed vector $\hat{v}$, denoted with mean squared error (MSE) which can be calculated by

(3) $$\begin{array}{c} \text{MSE}=E\left[d^{2}\left(v,\hat{v}\right)\right]=E\left[{\left\|x-\hat{x}\right\|}^{2}\right]. \end{array}$$

The smaller the MSE is, the better the codebooks are. The proposed accumulative quantization aims to minimize MSE in the process of training *L* codebooks and encoding vectors, respectively.

### 2.1. Codebook Training

Given a training vector set *X*={*x*_1_, *x*_2_,…*x*_*N*_}, *x*_*i*_ ∈ R^*d*^, accumulative quantization initially decomposes each training vector into *L* partial vector of the same dimension as that of original vector, where *x*_*i*_=∑_*i*=1_^*L*^*x*_*i*,*l*_.

Then, the training set is decomposed into *L* training partial vector sets *X*(*l*) ={*x*_*i*,*l*_}(*l*=1,2,…, *L*), where *x*_*i*,*l*_ denotes the *l*th partial vector of the vector *x*_*i*_.

Figure 1(a) shows the framework of codebooks training for proposed accumulative quantization, which consists of initial codebooks training and codebooks optimization.

#### 2.1.1. Initial Codebooks Training

To train the *L* initial codebooks, *k*-means algorithm is performed to generate *k* centroids as the codebook *C*_*l*_={*c*_*l*,1_, *c*_*l*,2_,…, *c*_*l*,*k*_} on training set *X*(*l*). Then, vector *x*_*i*_ can be quantized by these *L* codebooks independently after decomposing this vector into *L* partial vector *x*_*i*,*l*_ according to

(4) $$\begin{array}{c} {\hat{x}}_{i,l}=\arg\underset{c_{l,j}\in C_{l}}{\min}d\left(x_{i,l},c_{l,j}\right),\;\left(j=1,2,\ldots ,k\right). \end{array}$$

where ${\hat{x}}_{i,l}$ denotes the quantization output of the *l*th partial vector *x*_*i*,*l*_ and *d*(*x*_*i*,*l*_, *c*_*l*,*j*_) denotes the Euclidean distance between *x*_*i*,*l*_ and the *j*th centroid *c*_*l*,*j*_ in codebook *C*_*l*_.

According to formula (3), the training errors can be measured by the mean square Euclidean distance between *x*_*i*_ and its reconstructed one ${\hat{x}}_{i}$, which is formulized as

(5) $$\begin{array}{c} \text{MSE}=\frac{1}{N}\sum_{i=1}^{N}{\left\|x_{i}-{\hat{x}}_{i}\right\|}^{2}=\frac{1}{N}\sum_{i=1}^{N}{\left\|x_{i}-\sum_{l=1}^{L}{\hat{x}}_{i,l}\right\|}^{2}, \end{array}$$

where $x_{i}-\sum_{l=1}^{L}{\hat{x}}_{i,l}$ is denoted as *e*_*i*_, representing the overall quantization error of *x*_*i*_. Also, $x_{i}-\sum_{l=1}^{L}{\hat{x}}_{i,l}$  =  ∑_*l*=1_^*L*^*e*_*i*_(*l*), where *e*_*i*_(*l*) denotes the quantization error of partial vector *x*_*i*,*l*_ produced by *C*_*l*_.

#### 2.1.2. Codebooks Optimizing

The objective function of training each codebook above is to minimize the error between *x*_*i*,*l*_ and ${\hat{x}}_{i,l}$ in each subvector set, not the MSE in (5); thus, those *L* codebooks may not be the optimal solution for the whole vectors.

Here, a codebook optimization is designed in an alternative manner, in which each step updates one group of parameters with fixing the others.

*UpdateC*_*l*_. Fixing {*C*_*l*′_, *l*′ ≠ *l*} and {$\hat{X}\left(l{}^{\prime }\right),l{}^{\prime }=1,2,\ldots ,L$}, the problem is transformed into recomputing the centroids according to vectors $\left\{x_{i}-\sum_{l\prime \neq l}^{L}{\hat{x}}_{i,l{}^{\prime }}\right\}=\left\{{\hat{x}}_{i,l}+e_{i}\right\}$ for the objective of minimizing the MSE. For each vector ${\hat{x}}_{i,l}+e_{i}$, a naive solution is to use ${\hat{x}}_{i,l}+e_{i}$ itself as the new centroids, replacing the closest centroid with vector ${\hat{x}}_{i,l}+e_{i}$, so that its MSE can be reduced to 0. However, this strategy may result in significantly increasing number of centroids in *C*_*l*_, so it is not practical. Inspired from k-means, we design a mean mechanism to update each *c*_*l*,*i*_ in *C*_*l*_, where *c*_*l*,*i*_ is recomputed as the mean of vectors whose nearest centroid is *c*_*l*,*i*_. The formula is showed as

(6) $$\begin{array}{c} c_{l,i}=\frac{1}{N_{c_{l,i}}}\sum_{i=1,NN\left({\hat{x}}_{i,l}+e_{i}\right)=c_{l,i}}^{N}\left({\hat{x}}_{i,l}+e_{i}\right), \end{array}$$

where *N*_*c*_*l*,*i*__ denotes the number of vectors whose nearest centroid is *c*_*l*,*i*_.

*Update* $\hat{X}\left(l\right)=\left\{{\hat{x}}_{i,l}\right\}$ . After optimizing *C*_*l*_, with fixed {*C*_*l*′_, *l*′ ≠ *l*} and {$\hat{X}\left(l{}^{\prime }\right)$}, the *lth* codebook changes, so the quantization output of *X*(*l*) should be updated together. It can be easily seen that the quantization outputs of vectors in *X*(*l*) are independent of each other. Then, the optimization of $\hat{X}\left(l\right)$ can be decomposed into *N* suboptimization according to formula (7) with given fixed {*C*_*l*′_} and $\left\{\hat{X}\left(l{}^{\prime }\right),l{}^{\prime }\neq l\right\}$:

(7) $$\begin{array}{c} \arg\underset{{\hat{x}}_{i,l}}{\min}{\left\|x_{i}-\sum_{l{}^{\prime }=1}^{L}{\hat{x}}_{i,l{}^{\prime }}\right\|}^{2}. \end{array}$$

The codebooks are optimized in iterative manner. One iteration includes the optimization from the 1st to the *L*th codebook sequentially. When the objective function value MSE showed in formula (5) converges, the process of codebooks optimization ends.

### 2.2. AQ-Based Vector Quantization

Given a vector *v*, vector quantization is supposed to generate an L-tuple containing *L* centroids by accumulative quantization to approximate *v*. The indices (binary code) of those *L* centroids are used as the codes to represent input vector. It can be achieved by respectively selecting one centroid from each codebook *C*_*l*_(*l*=1,…, *L*) to minimize the overall quantization error ${\left\|v-\sum_{l=1}^{L}{\hat{v}}_{l}\right\|}^{2}$.

A natural way is to compare all the *L*-tuples and select the best one. However, for each codebook containing *k* centroids, there are *k*^*L*^ comparisons to gain the quantization output. This will greatly weaken the efficiency; thus, it is not practical.

We propose a vector quantization method for accumulative quantization, including 2 procedures: initial quantization and quantization output optimizing, showed in Figure 1(b).

The procedure of initial encoding quantizes *v* with *L* quantizers independently after decomposing *v* into *L* partial vectors. The procedure of quantization output optimizing uses the overall quantization error *e*_*v*_ to sequentially update the *l*′ th quantization output from *l*′=1 to *l*′=L with fixed *L* codebooks and the other *L*-1 quantization outputs.

#### 2.2.1. Initial Quantization

The vector *v* is firstly decomposed into *L* partial vectors {*v*_1_,…*v*_*l*_,…, *v*_*L*_}, where *v*=∑_*i*=1_^*L*^*v*_*l*_. Then, each accumulative vector *v*_*l*_ is quantized by corresponding quantizer *Q*_*l*_ according to formula (4). Consequently, the *L* quantization outputs $\left\{{\hat{v}}_{1},\ldots {\hat{v}}_{l},\ldots ,{\hat{v}}_{L}\right\}$ are obtained. Thus, *v* can be approximated by its reconstructed vector $\hat{v}=\sum_{l=1}^{L}{\hat{v}}_{l}$.

#### 2.2.2. Quantization Outputs Optimizing

Partial vector *v*_*l*_ is quantized for the purpose of minimizing the error between *v*_*l*_ and ${\hat{v}}_{l}$, which can be measured by ${\left\|v_{l}-{\hat{v}}_{l}\right\|}^{2}$. While promising, procedure (1) can simplify the process of quantizing *v*, but the reconstruct vector $\sum_{l=1}^{L}{\hat{v}}_{l}$ may not be the best one to approximate *v*. The reason lies in the fact that each ${\hat{v}}_{l}$ is obtained considering only minimizing the local quantization error, not the overall quantization error ${\left\|v-\sum_{l=1}^{L}{\hat{v}}_{l}\right\|}^{2}$ between *v* and its reconstructed one $\hat{v}$.

An iterative optimization is proposed to improve the *L*-tuple quantization outputs with the *L* codebooks as constant. Like optimizing codebooks, each ${\hat{v}}_{l}$ is also optimized in an alternative manner.

Optimize ${\hat{v}}_{l}$. Fixing the other *L*-1 quantization outputs ${\hat{v}}_{l\prime }\left(l\prime \neq l\right)$, the residual vector $v-\sum_{l\prime \neq l}^{L}{\hat{v}}_{l\prime }={\hat{v}}_{l}+e_{v}$ is computed and taken as the input of the *l*th quantizer. Then, it is quantized according to formula (4), so that the *l*th quantization output is updated under the condition of minimizing the overall quantization error.

The *L*-tuple quantization output is optimized iteratively from the 1st to *L*th sequentially. The iteration stops until the *L*-tuple quantization outputs do not change. Experiments show that the proposed vector encoding method can rapidly converge in a little number of iterations, showed in Figure 2. Lower quantization brings the benefit that vectors can gain better approximation with fixed *L* codebooks.

## 3. Fast Distance Computation

When performing ANN search, the distance between the query vector *q* and the vector *y*_*i*_ in database needs to be computed, where the quantization output ${\hat{y}}_{i}$ of *y*_*i*_ is denoted as *L*-tuple $\left\{{\hat{y}}_{i,1},\ldots {\hat{y}}_{i,l},\ldots {\hat{y}}_{i,L}\right\}$. Based on accumulative quantization, an asymmetric Euclidean distance computing is proposed to accelerate ANN search, which is showed in the following:

(8) $$\begin{array}{c} d^{2}\left(q,y_{i}\right)\approx d^{2}\left(q,{\hat{y}}_{i}\right)=d^{2}\left(q,\sum_{l=1}^{:L}{\hat{y}}_{i,l}\right),\\ ={\left\|q-{\hat{y}}_{i}\right\|}^{2}={\left\|q-\sum_{l=1}^{:L}{\hat{y}}_{i,l}\right\|}^{2},\\ ={\left\|q\right\|}^{2}-2\langle q,\sum_{l=1}^{:L}{\hat{y}}_{i,l}\rangle +{\left\|\sum_{l=1}^{:L}{\hat{y}}_{i,l}\right\|}^{2}. \end{array}$$

For query vector *q*, the term ‖*q*‖^2^ is a constant for all database vectors and does not affect the ANN search, so it does not need to be computed.

1. Evaluating the term $\langle q,\sum_{l=1}^{:L}{\hat{y}}_{i,l}\rangle$: the term $\langle q,\sum_{l=1}^{:L}{\hat{y}}_{i,l}\rangle$ can be transformed as $\sum_{l=1}^{L}\langle q,{\hat{y}}_{i,l}\rangle$. Then, the term $\langle q,{\hat{y}}_{i,l}\rangle$ can be obtained from a look-up table, in which the inner product between *q* and the *L* × *k* centroids is precomputed when *q* is submitted.
2. Evaluating the term ${\left\|\sum_{l=1}^{:L}{\hat{y}}_{i,l}\right\|}^{2}$: if it is computed online when a query vector is submitted, the ANN search time efficiency will be inevitabley decreased. While promising, evaluating ${\left\|\sum_{l=1}^{:L}{\hat{y}}_{i,l}\right\|}^{2}$ can be transformed into computing $\sum_{l=1}^{L}\sum_{l\prime =1}^{L}\langle {\hat{y}}_{i,l},{\hat{y}}_{i,l\prime }\rangle$ which can also be obtained by constructing *L*^2^/2 look-up tables of *k* × *k* size, but the computation cost is large [25]. Another way is to compute the length ${\left\|\sum_{l=1}^{:L}{\hat{y}}_{i,l}\right\|}^{2}={\left\|{\hat{y}}_{i}\right\|}^{2}$ of reconstructed vector ${\hat{y}}_{i}$ offline and store it in a look-up table when quantizing *y.* However, each database vector needs 4 bytes to store ${\left\|{\hat{y}}_{i}\right\|}^{2}$.

Here, a simple uniform scalar quantization is designed to encode ${\left\|\hat{y}\right\|}^{2}$ with several binary bits, named length bits. For example, if it is planned to take 1 byte to store ${\left\|{\hat{y}}_{i}\right\|}^{2}$, ${\left\|{\hat{y}}_{i}\right\|}^{2}$ can be quantized by 256 discrete scale values, where a scale value is selected to approximate ${\left\|{\hat{y}}_{i}\right\|}^{2}$ and its indices are used to denote it. In this case, the proposed uniform quantization for ${\left\|{\hat{y}}_{i}\right\|}^{2}$ can be displayed in the following:

(9) $$\begin{array}{c} \frac{\max\left\{{\left\|{\hat{y}}_{i}\right\|}^{2}\right\}\;\times \left[255\times \left({\left\|\hat{y}\right\|}^{2}/\max\left\{{\left\|{\hat{y}}_{i}\right\|}^{2}\right\}\;\right)+0.5\right]}{255}. \end{array}$$

where [·] transforms ${\left\|{\hat{y}}_{i}\right\|}^{2}$ into an integer value ranging from 0 to 255. This is performed when the database vectors are quantized offline and stored in a look-up table. In the experiments later, we will show the influence of length bits' choices on the ANN search accuracy.

## 4. Hypersphere-Based Filtration for Exhaustive ANN Search

Given a query vector *q*, the distance between *q* and the vectors in database will be computed according to formula (8) when performing exhaustive ANN search. Then, a distance sorting method is adopted over all the vectors to return close vectors of presetting number.

To reduce the number of vectors in distance sorting, a hypersphere can be constructed for each query vector *q* in vector space. An example in 2D space is showed in Figure 3. Only the vectors lying in the hypersphere are taken into distance sorting. The others are filtered by the hypersphere. Thus, the problem that remains is how to determine the radius for each hypersphere.

In accumulative quantization, each codebook partitions the dataset into *k* clusters with each centroid as the center. Then, the first *L*′ (1 ≤ *L*′ ≤ *L*) codebooks can be considered to partition the dataset into *k*^*L*′^ clusters. Each center is the sum vector of *L*′ centroids, where each centroid is selected from a codebook respectively. The vectors in a cluster are usually considered to be similar to the center vector, but this similarity between vectors may not be transitive. In Figure 3, although center *g* does not lie in the sphere, there still are dots lying in the sphere.

Here, based on the first *L*′ codebooks of AQ, *k*^*L*′^ cluster centers can be produced. Then, for a query vector *q*, *w* nearest cluster centers can be obtained based on the distances computed according to formula (8). Finally, the hypersphere can be constructed, where the corresponding radius is computed as follows:

(10) $$\begin{array}{c} {\text{radius}}_{q}=\frac{1}{w}\sum_{i=1}^{w}d\left(q,c_{q,i}\right), \end{array}$$

where *c*_*q*,*i*_ belongs to the set containing the *w* nearest cluster centers of *q*. *d*(*q*, *c*_*q*,*i*_) is computed according to formula (8). Only the vectors whose distances to query vector *q* are smaller than radius_*q*_ are put into sorting when performing exhaustive ANN search.

The granularity of partitioning dataset is finer if *L*′ is larger. Under fixed *L*′, the radius of hypersphere is larger with increasing *w*, which results in less vectors to be filtered by hypersphere.

## 5. Experiments

All the experiments are measured on a machine with Xeon 16 cores 2.4GHZ CPU and 16 GB RAM, except for the experiments on 1B SIFT with 256G RAM.

### 5.1. Datasets

Three publicly available datasets [4], SIFT descriptor dataset and GIST descriptor dataset, are used to evaluate the performance. SIFT descriptor codes small image patch while gist descriptor codes the entire image. SIFT descriptor is a histogram of oriented gradients extracted from gray image patch. GIST descriptor is similar to SIFT but applied to the entire image. It applies an oriented Gabor filter over different scales and averages the filter energy in each bin.

SIFT and GIST datasets have three subsets: learning set, database set, and query set. The learning set is used to train stage-codebooks, and the database and query sets are used for evaluating quantization performance and ANN search performance. For SIFT dataset, the learning set is extracted from Flicker images [28] and the database and query vectors are extracted from INRIA holidays images [29]. For GIST dataset, the learning set consists of the tiny image set of [30]. The database set is holidays image set combined with Flicker 1M [28]. The query vectors are extracted from the holidays image queries [29]. All the descriptors are high-dimensional float vectors. The details of datasets are given in Table 1.

### 5.2. Convergence of Training Codebook

In training codebook for accumulative quantization, the optimization aims to gain more accurate codebook, so that the vectors can be approximated more precisely when quantizing them. To implement this easily, instead of using a preset threshold, we set the total number of iteration (the total number is 20) as the convergence condition when optimizing codebooks for accumulative quantization. To evaluate the convergence of training codebook, this section shows the training error during codebook training on the 1M SIFT and 1M GIST, including initial codebook training and codebook optimization.

When decomposing each input vector *v* ∈ *R*^*d*^ into *L* partial vectors, *v* is firstly divided into *L* subvector of (*d*/*L*) dimension; then, each subvector is extended to *L* dimension by filling the other components with 0.

The parameter *L* representing the number of codebooks ranges within {4, 8, 12, 16}. The number of centroids in each codebook is set as the typical value *k* = 256.

In Figure 4, the iteration number 0 denotes the codebook training without codebooks optimization. As seen in Figure 4, the codebook optimization can obviously reduce the errors produced by initial codebooks training. Besides, the proposed codebook optimization can converge rapidly, which can be observed from the notion that the curves tend to be flat in less than 5 iterations on 1M SIFT dataset and 10 iterations on 1M GIST dataset. Then, the conclusion can be drawn that the codebook optimization can improve the approximation power of codebooks effectively.

### 5.3. Quantization Performance

Figure 2 shows the proposed vector quantization (vector encoding) mechanism converges rapidly. This section investigates the quantization performance of our approach through evaluating the overall quantization error measured by MSE between vectors and their reconstructed ones under different parameters: *k* and L. The code length nbits=*L*log_2_^*k*^ denotes the memory requirement to store a vector after quantizing it. K ranges within {16, 64, 256}, and *L* ranges within {4, 8, 12, 16}.

Figure 5 shows the trade-offs between overall quantization error and memory usage for a vector on 1M SIFT and 1M GIST. Generally, larger number of bits brings lower overall quantization error. Then, a vector is quantized more accurately. Besides, it can be observed from Figure 5 that the overall quantization error is reduced by increasing either parameter *k* or parameter *L*. Given a fixed number of bits, the proposed accumulative quantization with more centroids contained in each codebook and fewer number of quantizers can gain more accurate quantization output than that of fewer centroids contained in each codebook and larger number of quantizers. While promising, the former choice (larger *k* and smaller *L*) usually takes more time costs than the latter (smaller *k* and larger *L*) to quantize vector.

### 5.4. The Influence of Parameters on ANN Search Performance

To estimate the accuracy of the notion that vectors are approximated by their quantization outputs, exhaustive ANN search is implemented. Recall@R is used to measure the ANN search accuracy. Recall@R is defined as the proportion of query vectors for which the nearest neighbor is ranked in the first *R* position. The larger the recall@R is, the better the search accuracy is.

#### 5.4.1. The Influence of the Numbers *k* and *L*

Exhaustive ANN search is implemented based on the proposed AQ, in which the search time costs mainly consist of constructing look-up table and sorting candidates. For exhaustive ANN search, all the vectors in database are put into sorting. Then, the search time efficiency is mainly influenced by the time costs on constructing look-up table for each query vector.

Figure 6 shows the average ANN search time on 1M SIFT and 1M GIST under different *k* and *L*. The *k* ranges within {16, 64, 256, 512}, and the *L* ranges within {4, 8, 12, 16}. It can be seen that the average ANN search takes more time with increasing *k* or *L*. Under the same *L*, the larger the value of *k*, the more the computation needed in constructing each look-up table. Under the same *k*, the larger the value of *L*, the more the look-up tables needed to be constructed.

Figure 7 shows the exhaustive ANN search results by AQ on 1M SIFT and 1M GIST, using recall@100 to measure the search accuracy. Given *k* and *L*, the code length used to encode the vector is *L*log_2_^*k*^ bits. It can be seen that the search accuracy is improved with increasing *k* or *L*. Under the same code length, the search accuracy with large *k* and small *L* is better than that with small *k* and large *L*. On 1M SIFT, the recall@100 becomes 1 when code length is 96 bits.

On the trade-off between search accuracy and search time efficiency, Figures 6 and 7 show that it can be obtained if *k* = 256 and *L* = 8. Also, these settings of parameter values are the typical value provided in state-of-the-art reference. Then, we use typic *k* = 256 and *L* = 8 in followup experiments.

#### 5.4.2. The Influence of Length Bits

An asymmetric distance computing method is designed in formula (8) to accelerate distance computing between query vector and vectors in database when doing AQ-based ANN search. A uniform scale quantization is designed to quantize the third term ${\left\|\sum_{l=1}^{:L}{\hat{y}}_{i,l}\right\|}^{2}$ by using several binary bits, so that the requirement of storing the length is reduced when computing ${\left\|\sum_{l=1}^{:L}{\hat{y}}_{i,l}\right\|}^{2}$ offline. This section investigates the influence on ANN search under different number of length bits with *k* = 256 and *L* = 8. Conveniently, AQ denoted accumulative quantization-based ANN search by storing length of the third term, while AQ-n denotes using *n* bits to quantize the third term in formula (8).

Tables 2 and 3 show the exhaustive ANN search accuracy with AQ and AQ-*n* on 1M SIFT and 1M GIST datasets. The number of length bits determines the discrimination of the third term in formula (8). It is reflected by the fact that the search accuracy of AQ-*n* becomes more and more similar to AQ when increasing *n*. Due to larger dimensionality of GIST vector than SIFT vector, AQ-*n* needs more length bits to achieve the same search accuracy as AQ. It can be observed from Table 2 that AQ-8 and AQ own the same search accuracy on 1M SIFT dataset, while *n* need to be increased to 10 so that AQ-10 is comparable with AQ on 1M GIST.

#### 5.4.3. The Influence of Hypersphere Parameters

The hypersphere is constructed for each query to reduce the number of vectors putting into sorting, so that the ANN search time efficiency can be improved under the condition of no loss on search accuracy. This section evaluates the influence of *L*′ and *w* on the search performance. Parameter *L*′ denotes using centroids in the first *L*′ codebooks to build up *k*^*L*′^ (*k* and *L* are set as typical values 256 and 8, resp.) centers. Parameter *w* denotes getting *w* nearest centers from *k*^*L*′^ centers.

Figure 8 shows the search performance when applying hypersphere filtration in AQ-based exhaustive ANN search. By constructing a hypersphere for query vector, nonsimilar vectors can really be filtered so that only a part of vectors are taken into distance sorting, which can be observed from Figure 8. Compared to 1M GIST dataset, using hypersphere can filter more nonsimilar vectors on 1M SIFT dataset. Commonly, when *w* = 1, it gains the best effect on filtering nonsimilar vectors whether *L*' = 1 or 2 on both 1M SIFT and 1M GIST. Besides, it can be seen that the number of filtered vectors when *L*' = 2 is more than that when *L*' = 1. With increasing value *L*', the centers composed by the first *L*' codebook are more and more close to query vectors. Then, the constructed hypersphere by the *w* nearest centers becomes smaller, so that the number of vectors lying in the hypersphere will be reduced. Consequently, the number of filtered vectors increases.

The ANN search performance regarding recall@100 and search time cost per query vector is detailed in Table 4. By filtering vectors out of constructed hypersphere, the number of vectors taken into distance sorting is reduced, so that the search time cost can be decreased correspondingly. Moreover, the ANN search accuracy is not weakened compared to AQ without hypersphere filtration. It can be demonstrated that hypersphere filtration-based ANN search can improve search time efficiency without weakening the search accuracy.

### 5.5. Comparison with the State of the Art

We compare our approach with five state-of-the-art exhaustive ANN search methods: RVQ-based exhaustive search [18], ERVQ-based exhaustive search [28], PQ-based exhaustive search [4], CQ-based exhaustive search [25], and quarter product quantization-based exhaustive search [21], which are, respectively, indicated as RVQ, ERVQ, PQ, CQ, and QPQ. Correspondingly, our AQ-based exhaustive search method is indicated as AQ.

Those five methods typically set *k* = 256 and *L* = 8 in experiments, which is detailed, respectively, in references [4, 18, 21, 25, 28]; thus, we also use the same parameter settings in this experiment for consistency.

Figure 9 shows the comparison of exhaustive ANN search between our approach and those five ANN search methods on 1M SIFT and 1M GIST datasets, respectively. Recall@R is used to measure the ANN search accuracy, where *R* ranges within {1, 5, 10, 20, 50, 100}. For RVQ, ERVQ, and CQ, we use the typic value of parameters given in references, where *L* = 8 and stage centroids *k* = 256. Also, for PQ and QPQ, we use typic 64 bits to quantize the vectors, where each vector is divided into 8 subvectors and each subvector is quantized with codebook containing 256 centroids.

From Figure 9(a), it can be seen that AQ outperforms RVQ, ERVQ, PQ, and CQ under the same scale of codebooks, while AQ owns comparable ANN search accuracy with QPQ. However, QPQ uses 2 nearest centroids to approximate each subvector during quantization procedure. Then, each subvector needs to spend twice the number of bits to represent it compared to AQ. Consequently, under the same scale of codebooks, QPQ needs twice the memory compared to AQ to store the codes when quantizing vectors. Therefore, it can be observed that AQ can consume less memory than QPQ under the condition of obtaining the same recall@R.

On 1M GIST dataset, due to the structured characteristics of GIST vectors, there is a structured version of PQ by regrouping GIST vectors, named as S-PQ, while natural PQ denotes PQ without regrouping GIST vectors. The ANN search accuracy of QPQ and natural PQ decreases more significantly than the other methods.  Figure 9(b) shows the ANN search accuracy of AQ is superior to that of RVQ, ERVQ, S-PQ, QPQ, and natural PQ. Comparing the curves between AQ and CQ in Figure 9(b), AQ is inferior to CQ when *R* < 20, while AQ outperforms CQ when *R* > 20.

Tables 5 and 6 detail the search accuracy and time efficiency of exhaustive ANN search by the above 6 methods, where the efficiency is measured by runtime tested on our machine. Due to the lower dimensionality of vector in SIFT dataset, those methods performed on SIFT dataset can obtain better ANN search time efficiency than that on GIST dataset. The search time of PQ and QPQ is slightly less than that of RVQ, ERVQ, CQ, and AQ. The reason lies in the fact that PQ and QPQ use lower dimensional subvector to construct the look-up tables while the others use the whole vector. In ERVQ, the final number of centroids in each stage-codebook may be smaller than preset value *k*, so the ANN search time efficiency by ERVQ is slightly superior to RVQ, CQ, and AQ, while these 3 methods own almost the same ANN search time cost per query.

When AQ is combined with hypersphere filtration mechanism, the ANN search time efficiency is improved due to the reducing number of vectors put into sorting. Moreover, it can be observed from Tables 5 and 6 that the ANN search time efficiency of AQ with filtration is superior to that of other methods.

Table 7 shows the exhaustive ANN search performance comparison on 1B SIFT dataset. Similar to [25], the first 1M learning vectors are used for efficient codebooks training. It can be seen that AQ obtains the best recall@100 among those 6 methods. It means that the improvement on ANN search is consistent.

For exhaustive ANN search, it needs to compute the approximate distances from query vector to all the vectors in the database and then do sorting. Therefore, compared to Table 5, under the same condition, the performance on 1B SIFT dataset is worse than that on 1M SIFT dataset, especially taking much more search time, which is consistent for the other methods. It is reasonable as searching in larger number of vectors is more difficult.

## 6. Conclusions

In this paper, we present an accumulative quantization for approximate nearest neighbor search. It exploits the accumulation of centroids from several codebooks to approximate a vector. For this purpose, a codebook optimization is designed to improve the approximation ability of codebooks by minimizing the overall quantization errors. When encoding vectors offline, the quantization outputs are optimized iteratively to reduce quantization error. Thus, the proposed accumulative quantization can achieve superior approximate nearest neighbor search accuracy to the state of the art. A uniform scale quantization is designed to reduce the requirement of storing the norm of ${\left\|{\hat{y}}_{i}\right\|}^{2}$. Empirical results show that the search accuracy can be guaranteed with a small number of bits. A hypersphere-based filtration is proposed to reduce the number of vectors putting into sort on the condition of no influence on search accuracy. Experiments show that the search time efficiency can be improved towards natural search.

In the further work, we will investigate the efficient nonexhaustive ANN search with AQ.

## Figures and Tables

**Figure 1:** The framework of accumulative quantization. (a) Training *L* codebooks. (b) Quantizing an input vector *v*.

**Figure 2:** The convergence of our vector encoding method over a representative dataset of 1M SIFT features with 64 bits (8 codebooks and each codebook contains 256 centroids). The vertical axis represents the quantization error according to formula (5). The horizontal axis represents the number of iterations.

**Figure 3:** An example of constructing a hypersphere for query q in 2D space. The blue dots lying out of the sphere are filtered. The orange dots lying in the sphere are taken into sorting with distances to the query point.

**Figure 4:** The errors produced by training L codebooks on different dataset. (a) The training errors on 1M SIFT dataset. (b) The training errors on 1M GIST dataset.

**Figure 5:** The overall quantization errors associated with various *k* and *L*. (a) The overall quantization errors on 1M SIFT dataset. (b) The overall quantization errors on 1M GIST dataset.

**Figure 6:** Average ANN search time under different *k* and *L*. (a) Search time on 1M SIFT dataset. (b) Search time on 1M GIST dataset.

**Figure 7:** Exhaustive ANN search accuracy under different *k* and *L*. (a) The recall@100 on 1M SIFT dataset. (b) The recall@100 on 1M GIST dataset.

**Figure 8:** Performance of hypersphere filtration-based exhaustive ANN search under different *w* and *L*′. (a) Effects of filtering vectors on 1M SIFT. (b) Effects of filtering vectors on 1M GIST.

**Figure 9:** Comparison of exhaustive ANN search for ANN. (a) Recall@R of varying *R* on 1M SIFT dataset. (b) Recall@R of varying *R* on 1M GIST dataset.

**Table 1:** Summary of the used datasets.

Information	1M SIFT	1M GIST	1B SIFT
Dimension of vectors	128	960	128
Size of learning set	100,000	500,000	100,000,000
Size of database set	1,000,000	1,000,000	1,000,000,000
Size of query set	10,000	1,000	10,000

**Table 2:** ANN search accuracy on 1M SIFT.

Methods	Recall@1	Recall@10	Recall@100
AQ	0.30	0.74	0.98
AQ-6	0.29	0.72	0.97
AQ-7	0.30	0.74	0.98
AQ-8	0.30	0.74	0.98
AQ-9	0.30	0.74	0.98
AQ-10	0.30	0.74	0.98

**Table 3:** ANN search accuracy on 1M GIST.

Methods	Recall@1	Recall@10	Recall@100
AQ	0.11	0.35	0.74
AQ-8	0.09	0.28	0.60
AQ-9	0.10	0.33	0.70
AQ-10	0.11	0.35	0.73
AQ-11	0.11	0.35	0.73
AQ-12	0.11	0.35	0.74

**Table 4:** Exhaustive ANN search performance by AQ and its variants with hypersphere-based filtration.

Dataset	Methods	Recall@100	Search time (ms)	Sorting number
1M SIFT	AQ, no filtering	0.98	66.9	1M
	AQ, *L*' = 1, *w* = 1	0.98	44.3	371K
	AQ, *L*' = 2, *w* = 1	0.98	42.0	292k

1M GIST	AQ, no filtering	0.74	71.9	1M
	AQ, *L*' = 1, *w* = 1	0.74	68.1	809k
	AQ, *L*' = 2, *w* = 1	0.74	60.7	621k

**Table 5:** Comparison of ANN search on 1M SIFT.

Methods	Parameters	Search time (ms)	Recall@100
RVQ	*k* = 256, *L* = 8	67.1	0.94
ERVQ	*k* = 256, *L* = 8	65.2	0.96
PQ	*k* = 256, *n* = 8	63.1	0.92
CQ	*k* = 256, *L* = 8	66.2	0.97
QPQ	*k* = 256, *n* = 8	65.9	0.97
AQ (ours)	*k* = 256, *L* = 8	66.9	0.98
AQ with filtration (ours)	*k* = 256, *L* = 8 L' = 2, *w* = 1	42.0	0.98

**Table 6:** Comparison of ANN search on 1M GIST.

Methods	Parameters	Search time (ms)	Recall@100
RVQ	*k* = 256, *L* = 8	71.3	0.68
ERVQ	*k* = 256, *L* = 8	69.6	0.71
S-PQ	*k* = 256, *n* = 8	66.9	0.65
CQ	*k* = 256, *L* = 8	72.0	0.73
QPQ	*k* = 256, *n* = 8	68.3	0.38
AQ (ours)	*k* = 256, *L* = 8	71.9	0.74
AQ with filtration (ours)	*k* = 256, *L* = 8 L' = 2, *w* = 1	60.7	0.74

**Table 7:** Comparison of ANN search on 1B SIFT.

Methods	Parameters	Search time (s)	Recall@100
RVQ	*k* = 256, *L* = 8	62.6	0.68
ERVQ	*k* = 256, *L* = 8	61.2	0.69
PQ	*k* = 256, *n* = 8	58.3	0.58
CQ	*k* = 256, *L* = 8	61.7	0.70
QPQ	*k* = 256, *n* = 8	60.6	0.69
AQ (ours)	*k* = 256, *L* = 8	62.2	0.72
AQ with filtration (ours)	*k* = 256, *L* = 8 *L*' = 2, *w* = 1	47.1	0.72

## Data Availability

The data used to support the findings of this study are available from the corresponding author upon request.
